# Aucubin Exerts Anticancer Activity in Breast Cancer and Regulates Intestinal Microbiota

**DOI:** 10.1155/2022/4534411

**Published:** 2022-05-16

**Authors:** Min Shao, Ziyun Kuang, Wenlin Wang, Shengnan Li, Guizhen Li, Yu Song, Haitao Li, Guozhen Cui, Hefeng Zhou

**Affiliations:** Department of Bioengineering, Zhuhai Campus of Zunyi Medical University, Zhuhai, China

## Abstract

Aucubin, a natural compound isolated from herbal medicine, has been reported to possess multiple beneficial properties. In this study, we aimed to verify the anticancer effect of aucubin on breast cancer and investigate the effect of cancer on the intestinal flora and whether aucubin has a therapeutic effect on intestinal problems caused by cancer. We established the breast cancer model with mouse 4T1 cell line and BALB/c mice. Aucubin was given once a day by gavage for 14 days. The results showed that aucubin suppress the growth of tumor *in vivo* by inducing tumor cell apoptosis. The tumor suppression rate of aucubin could reach 51.31 ± 4.07%. Organ histopathology was evaluated by tissue staining, which demonstrated that aucubin could alleviate the organ inflammatory damage caused by breast cancer without visible side effects. Moreover, aucubin could increase the expression of colonic tight junction protein occluding and adjust the gut microbiome to normal level according to 16S rDNA high-throughput sequencing. Herein, our results provide evidence for developing aucubin as an alternative and safe therapeutic for breast cancer treatment.

## 1. Introduction

Breast cancer is the most common cancer diagnosed among women, and ranks among the most three common cancers worldwide, along with colon and lung cancers [1]. Due to the advancement of tumor surgery technology and neoadjuvant tumor reduction drug treatments [2], breast cancer without detectable distant metastases is considered curable in the early stages. The current mainstream treatment strategies include surgical resection, adjuvant chemotherapy, radiotherapy and hormone therapy, which are accompanied by severe adverse effects and respective limitations. Breast cancer can damage the intestinal barrier of patients [3], which may put the body into a dysregulated state and lead to disease initiation and progression. Adjuvant chemotherapy is often accompanied by serious gastrointestinal syndrome, such as intestinal inflammation and diarrhea, which can seriously limit the dosage and efficacy of drugs [4]. Therefore, the selection of ideal drugs in the process of tumor treatment is still being explored.

A research of gut microbiota difference between postmenopausal breast cancer case patients and control patients showed that statistically significantly differences exist in composition (*β*-diversity, *p*=0.006) [3]. Microbial metabolism of the gastrointestinal tract can regulate the development and function of the host immune system [5]. The microbial metabolism of drugs can affect the therapeutic effect, which may improve the treatment efficacy. Studies have shown that healthy gut flora may modulate responses to anti-programmed cell death ligand 1 immunotherapy in melanoma patients to help fight cancer [6, 7]. Moreover, microbial metabolism is found to be able to reverse the Warburg effect by increasing the levels of histone-acetylation and butyrate, which is helpful for suppressing tumors [8]. In some cases, gut microbiome metabolism can activate the mutation of the drug's toxicity to cause serious drug adverse effects, including severe diarrhea and life-threatening [9]. Therefore, making good use of the double-edged sword of gut flora is of great significance for cancer treatment.

Aucubin is an iridoid glycoside compound (Figure 1(a)) that is widely present in many plants, especially high in *Plantago asiatica*, *Eucommia ulmoides*, and *Aucuba japonica*. A series of studies have demonstrated that aucubin possess multiple beneficial effects including antioxidation [10, 11], anti-inflammation [12], anti-fibrosis [13], hepatoprotection [14], neuroprotection [15], osteoprotection [16], antitumor [17], antiendothelial dysfunction [18], and antiphotoaging [19]. Aucubin is a low toxic compound. Normal Wistar rats can still survive by a single intraperitoneal injection with 100 mg/kg dose of aucubin [20]. It has wide range of functions, low toxicity, and is not easy to cause secondary harm to cancer patients, making aucubin a very promising anticancer drug.

## 2. Materials and Methods

### 2.1. Chemicals and Reagents

Aucubin with purity over 95% was supplied by Chengdu Must Bio-Technology Co. Ltd. (Sichuan, China). Roswell Park Memorial Institute (RPMI) 1640, fetal bovine serum (FBS), antibiotic-antimycotic solution, penicillin/streptomycin, phosphate-buffered saline (PBS), and 0.25% (w/v) trypsin/1 mM EDTA were procured by Gibco (Thermo Fisher Scientific, USA). Annexin V-FITC Apoptosis Detection Kit was purchased from Elabscience Biotechnology Co. Ltd. (Hubei, China).

### 2.2. Cell Culture

Murine metastatic breast cancer 4T1 cell line was obtained from the American Type Culture Collection (ATCC, Manassas, VA). Cells were cultured in RPMI 1640 medium supplemented with 1% penicillin/streptomycin and 10% FBS, and maintained in incubators at 37°C under an atmosphere of 5% CO_2_.

### 2.3. Animal Models

The specific pathogen-free (SPF) female BALB/c mice (6 weeks old, 18–20 g) were purchased from the Guangdong Medical Laboratory Animal Center (China). Mice were housed in pathogen-free conditions (22 ± 2°C, 50 ± 5% humidity, 12 h light/dark cycle) with food and water freely to acclimatize for 7 days. All experiments involving animals were approved by Institutional Animal Care and Use Committee, Zunyi Medical University. To obtain the xenograft animal model, 4T1 cells (6 × 10^6^) were suspended in 60 *μ*L PBS and inoculated into the left flank of mice. When the palpable tumor volume increased to 50–100 mm^3^, mice were randomly divided into four groups and received different treatments. The schematic depicting of the animal model is shown in Figure 1(b). To evaluate therapeutic efficacy, tumor volume and body weight were measured every day. Tumor volume (*V*) was calculated based on equation (1), and tumor suppression rate (TSR) were calculated based on equation (2).

(1) $$\begin{array}{c} V=a\times \frac{b^{2}}{2}, \end{array}$$

(2) $$\begin{array}{c} \text{TSR}=\frac{\left(W_{c}‐W_{x}\right)}{W_{c}}\times 100\%. \end{array}$$

The largest diameter (*a*) and smallest diameter (*b*) of the tumors were measured with vernier caliper. *W*_*c*_ and *W*_*x*_ represent tumor weight of the model group and treatment group, respectively. The mice were sacrificed by cervical dislocation. The tumors and organs were excised and weighed, and quickly fixed in 4% paraformaldehyde for hematoxylin and eosin stains (H&E).

### 2.4. Tumor Cell Apoptosis

The tumor tissue was digested into a single cell suspension, and the cells were rinsed with PBS twice. 5 × 10^5^ cells were resuspended in 500 *μ*L 1× annexin V binding buffer, then 2.5 *μ*L of annexin V-FITC, and 2.5 *μ*L of PI staining solution were added and incubated at room temperature for 20 minutes in the dark. At last, 400 *μ*L diluted 1× annexin V binding buffer was added in the mixture. Cell apoptosis was detected by flow cytometry (Beckman Coulter, America).

### 2.5. Immunohistochemistry

The tumor was embedded in paraffin. The sample was sliced and then deparaffinized. The sample was immersed in citric acid antigen retrieval buffer for antigen retrieval. The slices were put in 3% hydrogen peroxide solution and incubated at room temperature without light for 25 min to block endogenous peroxidase. After washing with PBS, BSA was added dropwise on chamber slides and incubated for 30 min, and the primary antibody was added to incubate overnight at 4°C. Then, it was washed three times with PBS, and the secondary antibody was added and incubated for 50 min at room temperature. After washing with PBS, enhanced DAB solution was added dropwise. After staining the nucleus with Harris hematoxylin, samples were observed under microscope and images were collected.

### 2.6. Immunofluorescence Staining

The intestinal tissue was embedded in paraffin. The sample was sliced and then deparaffinized. Then, the sample was immersed in EDTA antigen retrieval buffer for antigen retrieval. BSA was added dropwise on chamber slides and incubated for 30 min, and the primary antibody was added to incubate overnight at 4°C. After washing three times with PBS, the secondary antibody was added and incubated for 50 min at room temperature without light. After washing with PBS, antifluorescence quenching solution was added dropwise. Samples were observed under a fluorescence microscope, and images were collected.

### 2.7. Serum Biochemical Test

The mice blood was collected in a sterile clean, enzyme-free EP tube by orbital blood collection, left it at room temperature for 20 minutes, and then centrifuged at 3000 r/min for 5 minutes. The upper serum was collected in a new sterile clean, enzyme-free EP tube and BCA method was used for protein quantification. The content of aspartate aminotransferase (AST) and alanine transaminase (ALT) in the serum was detected by using the automatic biochemical analyzer (Mindray, China).

### 2.8. 16S rDNA High-Throughput Sequencing Bioinformatics Analysis

About 100 mg of intestinal contents were taken from each mouse, and microbial community genomic DNA was extracted with the E.Z.N.A.® soil DNA Kit (Omega Bio-tek, Norcross, GA, USA). After PCR amplification, the pure DNA product is harvested by using the AxyPrep DNA Gel Extraction Kit (Axygen Biosciences, Union City, CA, USA). Purified amplicons were pooled in equimolar and paired-end sequenced on an Illumina NovaSeq PE250 platform (Illumina, San Diego, USA) according to the standard protocols by Majorbio Bio-Pharm Technology Co. Ltd. (Shanghai, China). Raw 16S rRNA gene sequencing reads were demultiplexed, quality-filtered by fastp version 0.20.0 [21] and merged by FLASH version 1.2.7 [22]. The sequences were grouped into provisional clusters as amplicon sequencing variants (ASVs). The taxonomy of each ASV representative sequence was analyzed by RDP Classifier version 2.2 [23].

### 2.9. Statistical Analysis

The GraphPad Prism 6.0 statistical software (San Diego, CA) was used for statistical analysis. The results were shown as mean ± standard deviation (SD). Statistical significance was assessed by one-way ANOVA followed by Tukey's multiple comparison, and *p* < 0.05 was considered as a statistical difference.

## 3. Results and Conclusion

### 3.1. Aucubin Suppressed the Growth of Tumor *In Vivo*

The mouse 4T1 cell line and BALB/c mice were used to establish the breast cancer model. When the palpable tumor volume increased to 50–100 mm^3^, mice were randomly divided into four groups (*n* = 6): (1) water, (2) 50 mg/kg of aucubin, (3) 100 mg/kg of aucubin, and (4) 200 mg/kg of aucubin. Drugs were given once a day by gavage.

The BALB/c mice without receiving inoculation of 4T1 cells were set as the control group treat with water. Tumor volume and body weight were measured every day to evaluate the therapeutic efficacy. There was no significant difference in the body weight of the mice in all groups after 14 days of continuous monitoring (Figure 1(c)).

As model group, the tumor of water increased faster from the 8th day and reached to 877 mm^3^ at day 14 (Figure 2(b)). In terms of tumor weight (Figure 2(c)), the group with drug treatment significantly inhibited the growth of tumors. The TSR of 50 mg/kg of aucubin, 100 mg/kg of aucubin, and 200 mg/kg of aucubin were 37.44 ± 8.71%, 51.31 ± 4.07%, and 50.34 ± 6.37%, respectively. We have also noticed that when the dose of aucubin is less than 100 mg/kg, the inhibitory effect on tumors increases with the gain of the dose. When the dose is greater than 100 mg/kg, there was no better or worse effect. The effect on the induction of apoptosis by aucubin on the tumor was presented in Figure 2(d). Compared with the model group, the percentage of the early and late apoptotic cells all significantly increased in the administration group. When the concentration increased to 100 mg/kg, the percentage of the total apoptotic cells increased to 58.67 ± 5.83%.

We performed H&E histological staining of the tumor tissue to observe cytopathological features (Figure 2(e)). In the model group, tumor cells are tightly arranged and mitosis is very common. The administration group, a large area of pink cytoplasm and prominent nuclear chromatin condensation could be clearly seen, demonstrating that cell proliferation is inhibited. The results of Ki67 and TUNEL assay also supported this conclusion (Figure 2(f)). Ki67 was expressed in large amounts in tumor tissues of the model group, which indicating that the cells proliferated vigorously. On the contrary, TUNEL was highly expressed in tumor tissues of the administration group. All these data might indicate that aucubin can inhibit tumor growth by inducing cell apoptosis.

### 3.2. Aucubin Showed No Harm to the Vital Organs of Mice

In order to analyze whether aucubin would have some side effects on mice, we detected the body weight, serum biochemical indexes, weight, and cytopathological features of vital organs. As present in Figure 3(a), compared with the control group, breast cancer tumors have no significant effect on the heart and kidneys weight of mice. However, it can cause significant inflammatory enlargement of the lung and spleen. Aucubin can improve this symptom, and low-dose of aucubin shows better effect. Although the protective effect of aucubin on the liver is not clearly reflected in the liver weight, it reduces the concentration of AST in the serum of mice (Figure 3(b)), indicating that it has a protective effect on the liver.

According to the H&E histological staining result (Figure 3(c)), we found that breast cancer can cause inflammation and tissue damage in vital organs. Aucubin has not been found to cause additional discernible damage to the organs. To a certain extent, aucubin helps the organs to recover to a normal state, which helps reduce inflammation and bleeding problems. Maintaining the integrity of the intestinal tract is the prerequisite for achieving the intestinal barrier function. Comprehensive detection of H&E and immunofluorescence staining (Figure 3(d)) on colon, we found that breast cancer can decrease the depth of colonic crypts and reduce the expression of tight junction protein occludin. In aucubin-treated mice with high doses, there was obvious increase of colonic occludin expression as can be seen by increase in occludin staining (green).

### 3.3. Effect of Aucubin on Breast Cancer-Induced Gut Dysbiosis

18 samples of fecal from three groups (control, model, and 100 mg/kg of aucubin) were collected, and we compared the gut microbiota of mice in different groups using 16S ribosomal RNA (rRNA) gene amplicon sequencing. The sequences were grouped into provisional clusters as ASV and analyzed on the Illumina NovaSeq PE250 platform. The *β*-diversity was reflected through principal co-ordinates analysis (PCoA).  Figure 4(a) shows that there was a significant distance between the intestinal flora of the groups, especially between groups control and model, which means that the occurrence of breast cancer can induce significant changes in the intestinal flora of mice. The taxon abundance of each sample was finally classified into 14 phyla and 217 genera (Figure 4(b)). Firmicutes, Bacteroidetes, and Deferribacteres were three major phyla in the gastrointestinal microbiota. The proportion of them in the gut has a significant difference between the groups. However, the proportions in the aucubin group are between group control and model, which indicating that aucubin can alleviate the changes in the intestinal microbiota caused by breast cancer. Linear discriminant analysis effect size (LEfSe) also proves that aucubin would not cause great unnormal effects on the intestinal flora. LEfSe can help us to find the species characteristics that best explain the differences between the three groups of samples, as well as the degree of influence of these characteristics, and obtain significantly different species. The blue node in cladogram (Figure 4(c)) indicates that the microbial group is enriched in the aucubin group, and there are only six of them.

According to the one-way ANOVA bar plot at the family level (Figure 4(d)), *Lactobacillaceae* and *Bacillaceae* in the model group are significantly decreased. On the contrary, *Staphylococcaceae*, *Bacteroidaceae*, and *Muribaculaceae* exhibited higher abundance. The aucubin group shows the ability to adjust the gut microbiome to normal level. Aucubin could increase the reduction in the proportion of microflora due to tumors, such as *Lachnospiraceae*, *Lactobacillaceae, Bacillaceae*, and *Ruminococcaceae*. It could also reduce the increase in the proportion of microflora, such as *Muribaculaceae, Staphylococcaceae*, *Oscillospiraceae, Bacteroidaceae, Marinifilaceae, Precotellaceae*, and *Tannerellaceae.* The KEGG ortholog functional profile level of the microbial community is predicted by PICRUSt based on 16S rRNA sequencing data, which is shown in Figure 4(e). The abundance of the KEGG-related pathway in the model group is generally lower than control and aucubin group, such as microbial metabolism in diverse environment, biosynthesis of amino acids and ribosome. The aucubin group shows the ability to adjust most of this pathway to normal level.

## 4. Discussion

Breast cancer without detectable distant metastases is considered curable in the early stages. The selection of ideal drugs in the process of tumor treatment is still being explored. Aucubin is a safe natural compound which is isolated from herbal medicine. A long-term toxicity study shown that oral administration of 200–800 mg/kg of aucubin had no significant effect in normal rats [24]. According to the breast cancer model with mouse 4T1 cell line and BALB/c mice, aucubin was shown to inhibit the growth of tumor *in vivo* by inducing tumor cell apoptosis. The tumor suppression rate of aucubin could reach 51.31 ± 4.07%.

Hepatotoxicity is one of the main side effects of cancer chemotherapy, including steatosis, pseudocirrhosis, long-term hepatic damage, cirrhosis, and even hepatic necrosis. It is previously reported that aucubin was mainly distributed to the kidney and liver [25]. It could reduce the generation of reactive oxygen species stimulated by TGF-*β*1 through suppressing the activity of NOX4. The antioxidative activity of aucubin contributed much to its hepatoprotection [14]. In the present work, we found that aucubin could decrease the concentration of AST in the serum of mice, which further indicated the hepatoprotective effect of aucubin. Aucubin was shown to alleviate the organ inflammatory damage during breast cancer progression. Combined with serum biochemical indicators and H&E histological staining result, it was found that these indicators tended to be close to the normal group.

A complication of cancer is that the intestinal flora disorder causes body weight loss and decreased immunity. Breast cancer has been widely reported to disrupt intestinal flora, which promotes tumor cell dissemination, metastatic seeding, and significant early inflammation through signaling in the gut [26, 27]. According to 16S ribosomal RNA (rRNA) gene amplicon sequencing and immunofluorescence staining on colon, aucubin has shown the ability to modulate the gut microbiome to normal level without chaos of other flora and increase the expression of colonic tight junction protein. A health intestinal barrier can help the drug to be absorbed and regulate the development and function of the host immune system. As dysregulated gut microbiota and intestinal barrier functions are highly associated with systemic diseases, aucubin may be a good choice for the treatment of other inflammatory diseases. Overall, understanding the ligand or mechanism of aucubin's effects on the human breast cancer cells is suggested for the future studies. The optimal mode of administration and dosage also warrants further study.

## 5. Conclusion

In conclusion, our study clearly verified the anticancer effect of aucubin on breast cancer in mouse model. We also found that aucubin has a therapeutic effect on intestinal problems by regulating intestinal microbiota. This research suggests that aucubin could be a promising anticancer compound in the breast cancer treatment and other diseases related to intestinal dysbacteriosis.

## Figures and Tables

**Figure 1:** Experimental design and the body weight of mice. (a) Chemical structure of aucubin. (b) The process of animal experiment. (c) The daily body weight changes of mice in different groups. Each value was expressed as the mean ± SD (*n* = 6 per group).

**Figure 2:** The antitumor activity of aucubin in vivo. (a) Excised tumors from tumor-bearing BALB/c female mice on the day after the last gavage. (b) The daily tumor volume changes of mice measured with vernier caliper in different groups. (c) Tumor weight of mice in different groups. (d) Cell apoptosis assay distribution of tumors. (e) H&E histological staining of tumor tissue from different groups. (f) Immunohistochemical staining of the Ki67 and TUNEL assay of tumor tissue from different groups. Each value was expressed as mean ± SD (*n* = 6 per group. ^*∗∗∗*^*p* < 0.001). Scale bars = 100 *μ*m.

**Figure 3:** The effect of aucubin on the vital organs of mice. (a) The weight of heart, liver, spleen, lungs, and kidneys from different groups. (b) The level of AST and ALT in serum from different groups. (c) Representative H&E staining of heart, liver, spleen, lungs, kidneys, and colon from different groups. (d) Immunofluorescence staining of colon ZO-1 (red) and occludin (green). Each value was expressed as mean ± SD (*n* = 6 per group. ^*∗*^*p* < 0.05, ^*∗∗*^*p* < 0.01, and ^*∗∗∗*^*p* < 0.001). Scale bars = 100 *μ*m.

**Figure 4:** The effect of aucubin on gut dysbiosis. (a) PCoA of the gut microbiome composition of mice on the ASV level at different groups. (b) Relative abundance at the phylum and genus level. (c) LEfSe multilevel species cladogram. (d) One-way ANOVA bar plot of family difference. (e) Comparison of PICRUSt-predicted relative abundance of KEGG pathway in different groups. Each value was expressed as mean ± SD (*n* = 6 per group). (^*∗*^*p* < 0.05 and ^*∗∗*^*p* < 0.01).

## Data Availability

The in vivo and in vitro data used to support the findings of this study are available from the corresponding author, Dr. Hefeng Zhou, upon request.
